# Modulation of the Pentose Phosphate Pathway Induces Endodermal Differentiation in Embryonic Stem Cells

This article has been retracted.

**DOI:** 10.1371/journal.pone.0029321

**Published:** 2012-01-12

**Authors:** Genesia Manganelli, Annalisa Fico, Ugo Masullo, Fabiana Pizzolongo, Amelia Cimmino, Stefania Filosa

**Affiliations:** 1 Stem Cell Fate Lab, Institute of Genetics and Biophysics “A. Buzzati Traverso” CNR, Naples, Italy; 2 IRCCS Neuromed, Pozzilli, Italy; 3 Faculty of Agriculture, University of Naples Federico II, Portici, Naples, Italy; Laurentian University, Canada

## Abstract

Embryonic stem (ES) cells can differentiate *in vitro* into a variety of cell types. Efforts to produce endodermal cell derivatives, including lung, liver and pancreas, have been met with modest success. Understanding how the endoderm originates from ES cells is the first step to generate specific cell types for therapeutic purposes. Recently, it has been demonstrated that inhibition of Myc or mTOR induces endodermal differentiation. Both Myc and mTOR are known to be activators of the Pentose Phosphate Pathway (PPP). We found that, differentely from wild type (wt), ES cells unable to produce pentose sugars through PPP differentiate into endodermal precursors in cell culture conditions generally non-permissive to generate them. The same effect was observed when wt ES cells were differentiated in presence of chemical inhibitors of the PPP. These data highlight a new role for metabolism. Indeed, to our knowledge, it is the first time that modulation of a metabolic pathway is described to be crucial in determining ES cell fate.

## Introduction

Endoderm-derived organ diseases include cystic fibrosis, chronic hepatitis, and diabetes; they affect more than 150 million people worldwide. Existing transplantation-based therapies are currently limited by the availability of donor-derived tissues.

Embryonic stem (ES) cells have the potential to give rise to any of the hundreds of cell types in the human body, raising exciting new prospects for biomedical research and for regenerative medicine [1]. Indeed, ES cells are a promising, renewable source of material for transplantation, because they can be expanded indefinitely in culture and can differentiate into all cell types of the body. Researchers are now taking advantage of the understanding of endoderm organogenesis to successfully direct the differentiation of ES cells into pancreas, liver, lung and thyroid cells [2]. The potential to virtually generate any differentiated cell type from ES cells offers the possibility to establish new models of mammalian development and to create new sources of cells for regenerative medicine. To realize this potential, it is essential to be able to control ES cells differentiation and to direct the development of these cells along specific pathways [1]. The molecular events regulating the induction and tissue-specific differentiation of endoderm are central to our understanding of the development and function of many organ systems [3].

Myc transcription factor and mTOR (Mammalian Target of Rapamycin) are both key regulators of cell growth and proliferation, and both have been described to control ES cells fate. In particular, Myc and mTOR repress endoderm differentiation of ES cells [4], [5]. Furthermore, both mTOR and Myc regulate the Pentose Phosphate Pathway (PPP). Indeed, it has been described that mTOR complex 1 activation leads to induction of genes encoding the enzymes of the PPP [6] and cMyc induces the production of ribose sugars, the product of the PPP [7].

We have generated mouse ES cells with a *G6pd* gene deletion (*G6pdΔ*). G6PD is the first and key enzyme of the PPP that, oxidizing glucose-6-phosphate, produces NADPH and pentose sugars. We have previously shown that these cells are extremely sensitive to oxidative stress, in keeping with the notion that G6PD is essential for production of high levels of NADPH, required for detoxification of reactive oxygen species [8], [9], [10], [11]. In addition, it has been reported that severe G6PD deficiency is lethal for mouse embryo. Severely G6PD-deficient hemizygous male embryos stop growing between E7.5 to E8.5 and show severe abnormalities, indicating that the role of G6PD is quite basic in mammalian development [12].

In this report we show, using engineered ES cells, that modulation of the PPP is necessary to drive ES cells differentiation into endodermal precursor cells. The data were confirmed in wt ES cells using two chemical inhibitors of the PPP. Moreover, we show that the mechanism does not involve the role of the PPP in providing reducing equivalent but rather its function in the production of pentose sugars.

## Results

### Analysis of gene expression during wt and *G6pdΔ* ES cells differentiation

We differentiated wt and *G6pdΔ* ES cells, using the previously described protocol to differentiate ES into neuronal cells [13], and analyzed the expression profiles of undifferentiated cells and three germ layers specific markers. As shown by RT-PCR, after 6 days of differentiation the expression of Oct4 and Nanog, markers of undifferentiated ES cells, are undetectable in both cell lines (Figure 1A). Moreover, no differences in the expression profile of Nestin (neuronal precursor marker), NF-L (marker of neurons), GFAP (glial cell marker), and Nkx2.5 were observed between wt and *G6pdΔ* ES cells (Figure 1A); αMHC (cardiomyocyte specific marker) and TDO (hepatocyte specific marker) were not expressed in both cell lines (data not shown). Instead, whereas endoderm was never formed during wt ES differentiation, from day 8 of differentiation in *G6pdΔ* ES cells we observed the expression of GATA4 (mesendodermal marker) and Sox17 (endodermal precursor marker) (Figure 1A). The expression of Sox17 was confirmed by immunofluorescence analysis on wt and *G6pdΔ* ES cells at 10 days of differentiation using anti-Sox17 antibody (Figure 1B). Since GATA4 was previously seen expressed in neurons and astrocytes [14], we analyzed, by immunofluorescence, the co-expression of GATA4 with βIII-tubulin (neural marker) or GFAP and we never observed co-expression of these markers (Figure S1A, B). Sox17 has been described to be expressed also in oligodendrocytes [15]; by western blot, we analyzed the expression of Olig2 (oligodendrocytes specific marker), but our cell culture method does not allow the differentiation of oligodendrocytes (Figure S1C). These data strengthen our hypothesis that GATA4 and Sox17 are expressed in endodermal precursors during *G6pdΔ* ES cells differentiation.

**Figure 1:** Endodermal induction in *G6pdΔ* ES cells. (A) Analysis of different markers in wt and *G6pdΔ* ES cells during neural differentiation. Expression profiles of undifferentiated ES cells (Oct4 and Nanog), neural precursors (Nestin), neurons (NF-L), astrocytes (GFAP), mesendodermal precursors (GATA4), endodermal precursors (Sox17), and cardiac precursors (Nkx2.5) markers were analyzed by RT-PCR. RNA was isolated from cells at different days of differentiation. Lane C, positive control, RNA isolated from 14dpc embryos. Amplified HPRT is shown as a positive control. (B) Double immunostaining Sox17/βIII-tubulin/DAPI of cells at 10 days of differentiation showed areas of immunoreactive cells for Sox17 only in *G6pdΔ* ES cells. Scale bars, 50 µm. (C) RT-PCR analysis of GATA4, Sox17, NF-L (neural marker), TH (dopaminergic neuron marker) and GAD65 (gabaergic neuron marker) on wt, two different *G6pdΔ* ES cell lines, and *G6pdΔ* ^pG6pd^ during differentiation. Lane C, positive control, on RNA isolated from 14dpc embryos. Amplified HPRT is shown as a positive control. (D) Western blot analysis with anti-Cripto and anti-Actin antibodies performed on protein extracts from wt and *G6pdΔ* ES cells during neural differentiation. Actin was analyzed as loading control. Below each lane the relative quantities (RQ) with respect to related undifferentiated embryonic stem cells are indicated. (E) Western blot analysis with anti-phospho-Smad2 and anti-Actin antibodies performed on protein extracts from wt and *G6pdΔ* ES cells during neural differentiation. Actin was analyzed as loading control. Below each lane the relative quantities (RQ) with respect to related undifferentiated embryonic stem cells are indicated.

To verify that the expression of endodermal specific markers was caused by inactivation of *G6pd* gene, and not by accidentally produced abnormalities, we confirmed, after differentiation, the expression of those markers in two different ES cell lines, *G6pdΔ1 and G6pdΔ2*, carrying the deletion of *G6pd* gene (Figure 1C). Moreover, in *G6pdΔ* ^p*G6pd*^ ES cells, *G6pdΔ* ES cells transfected with an expression vector containing a puromycin resistance gene in which the expression of *G6pd* is driven by the β-actin promoter [11], we never observed the expression of GATA4 and Sox17 (Figure 1C) although they differentiate in neuronal cell lines as proved by the expression of specific neuronal markers.

Nodal signalling participates in the nervous system patterning but also in mesendoderm induction. Smad2 is an essential intracellular transducer of the Tgf-β/Nodal signal. Nodal signalling through type I (ALK4 and ALK7) and type II (ActRIIA and ActRIIB) receptors in conjunction with its co-receptor, Cripto, is crucial for generating mesendoderm precursor cells. Following the engagement of Nodal with its receptor, Smad2 becomes phosphorylated and induces mesendodermal differentiation [16], [17], [18]. During differentiation we confirmed that Nodal was expressed both in wt and *G6pdΔ* ES cells although at higher level in the last one (Figure S1D). We also analyzed Cripto expression in wt and *G6pdΔ* ES cells. Although Cripto is already switched off at day 4 of differentiation in wt ES cells, its expression is still present at day 6 of differentiation in *G6pdΔ* ES cells (Figure 1D, Figure S1E). Moreover, we found that Smad2 phosphorylation is induced in differentiating *G6pdΔ* compared to wt until day 6 of differentiation, although this pathway is active also in wt ES cells during neuronal differentiation (Figure 1E).

### Induction of Definitive and Extraembryonic Endoderm

Sox17 is expressed in definitive endoderm but also in extraembryonic endoderm. Borowiak et al. (2009) found that Sox17+ cells can have two distinct morphologies: as dispersed Sox17+ cells or clustered populations [19]. They demonstrated that the dispersed Sox17+ cells also expressed extraembryonic endoderm markers. Positive identification of definitive endoderm is hindered by lack of unique markers that are expressed exclusively in these cells. Borowiak et al. (2009) concluded that clustered populations of Sox17+ cells are definitive endoderm, indeed these cells do not express extraembryonic markers [19]. Although we used a different protocol to differentiate *G6pdΔ* ES cells, we observed Sox17+ cells with both clustered and dispersed morphologies (Figure 2A). These data let us hypothesize that both extraembryonic and definitive endodermal cells could be differentiated from *G6pdΔ* ES cells.

**Figure 2:** Definitive and extraembryonic endoderm differentiated from *G6pdΔ* ES cells. (A) Immunofluorescent staining of the differentiated mouse *G6pdΔ* ES cells for Sox17 (red) and nuclei (blue) at 8 days of neural differentiation. PH, phase contrast images. Scale bars, 25 µm. (B) RT-PCR analysis of the endodermal markers GATA4 and extraembyonic endodermal markers Sox7 during differentiation. Lane C, positive control, RNA isolated from embryos and yolk sacs at 9,5 dpc. Amplified HPRT is shown as a positive control. (C) qRT-PCR for Pdx1 in wt and *G6pdΔ* ES cells at 13 days after treatment with Indolactam V from day 8 during differentiation. Values are means ± SD (n = 2). *P<0.05; **P<0.01; ***P<0.001.

To better define whether both cell populations are formed during *G6pdΔ* ES cell differentiation, we confirmed the presence of extraembryonic marker Sox7 by RT-PCR analysis (Figure 2B) [20]. Moreover, Chen et al. (2009) identified a small molecule, Indolactam V, that can induce differentiation of endodermal precursor cells (Sox17+) into pancreatic progenitor cells [21]. Wt and *G6pdΔ* ES cells at 8 days of differentiation were grown for 5 more days in presence of Indolactam V; the analysis by real-time RT-PCR (qRT-PCR) of mRNA extracts from both cell lines revealed the presence of Pdx1, a marker of pancreatic progenitors, exclusively in *G6pdΔ* ES cells (Figure 2C).

The presented data support our hypothesis that both extraembryonic and definitive endoderm Sox17+ cells are induced during *G6pdΔ* ES cells differentiation.

### Analysis of the mechanism inducing endodermal cell differentiation

Redox status mediates ES differentiation [22]. G6PD, a NADPH-producing dehydrogenase, is an enzyme essential for the defense of the cells against oxidative stress. To analyze whether oxidant formed in absence of G6PD have a role in establishing the mechanism that drives differentiation of *G6pdΔ* ES cells into endodermal cells, we differentiated wt and *G6pdΔ* ES cells with the previously described protocol in presence of a lower oxygen concentration described to be a physiological oxygen level during development (normoxia) [23], 5% instead of the 20% used in the normal culture conditions. Although in these culture conditions a reduced amount of ROS is formed (Figure S2A), we observed expression of GATA4 and Sox17 indicating that endodermal precursor cells are still differentiated (Figure 3A). Moreover, differentiating ES cells in presence of N-acetylcysteine (NAC), a well-known antioxidant molecule, *G6pdΔ* ES cells are still able to differentiate into endodermal cells, in fact they expressed GATA4 and Sox17, differently from wt ES cells (Figure S2B).

**Figure 3:** Mechanism inducing endodermal cell differentiation. (A) RT-PCR of different lineage-specific marker genes in wt and *G6pdΔ* ES cells in presence of a lower oxygen concentration (5%) and in normal culture conditions (20%). (B) RT-PCR of different lineage-specific markers in differentiated wt E14 and *Pgd*+/− ES cells at 8, 10 and 13 days of neural differentiation. (C) Double immunostaining Sox17/βIII-tubulin/DAPI of cells at 10 days of differentiation showed areas of immunoreactive cells for Sox17 only in *Pgd*+/− ES cells. Scale bars, 75 µm. (D) qRT-PCR for Sox17 and GATA4 in wt and *G6pdΔ* ES cells at day 10 after treatment with D-(-)-ribose during neural differentiation. Values are means ± SD (n = 3). *P<0.05; **P<0.01; ***P<0.001.

Being the first and key enzyme of the PPP, G6PD is essential also for the production of pentose sugars. To analyze whether the pentose sugars have a role in establishing the differentiation fate of *G6pdΔ* ES cells into endodermal precursors, we differentiated heterozygous knockout ES cells for Phosphogluconate Dehydrogenase (*Pgd*+/− ES cells), the second enzyme of the PPP, using the previously described protocol. These cells, compared to wt ES, have a reduced amount of *Pgd* mRNA (Figure S3A), a reduced flow of glucose carbon through the oxidative arm of the PPP (Figure S3B) and moreover, differently from *G6pdΔ* ES cells, they are not sensitive to oxidative stress (Figure S3C). As previously observed in *G6pdΔ*, also *Pgd*+/− ES cells are able to differentiate into endodermal cells (Figure 3B, C, Figure S3D, E, F). These data suggest that modulation of the PPP is important to drive endodermal fate.

Moreover, to confirm the hypothesis that the amount of pentose sugars present in the cells can influence the differentiation fate, we differentiated wt and *G6pdΔ* ES cells in presence of D-(-)-ribose. Although the addition of D-(-)-ribose had no effect on wt ES cells differentiation, we observed a reduction in the amount of Sox17 mRNA in *G6pdΔ* differentiated ES cells (Figure 3D), confirming our hypothesis. We observed the same effect differentiating *G6pdΔ* ES cells in presence of L-(-)-ribose, in contrast, addition of other sugars like L-Arabinose or Sucrose had no effect on Sox17 mRNA (Figure S3G)

The addition of D-(-)-ribose during differentiation to *G6pdΔ* ES cells had no effect on carbon flow through Glycolysis and citric acid cycle, Maillard reaction and did not increase the amount of ROS (data not shown).

### Chemical inhibitors of the PPP induce wt ES cells to differentiate into endodermal cells

DHEA and 6AN have been described to inhibit respectively G6PD and PGD activity [24], [25]. To confirm that DHEA and 6AN were inhibiting the PPP in ES cells, we measured, in wt ES cells the flow of glucose carbon through the oxidative arm of the PPP, at maximum non toxic concentration of both substances (DHEA and 6AN) and observed a statistically significant reduction of the pathway (Figure 4A); moreover, to verify that DHEA was acting on G6PD while 6AN was acting on PGD, we tested the capability to respond to oxidative stress of treated cells compared to wt and we observed that, as expected, DHEA treated wt ES cells were more sensitive to oxidizing agents as *G6pdΔ* ES cells [10], while 6AN treated cells show the same resistance as wt and *Pgd*+/− ES cells (Figure S4B).

**Figure 4:** Inhibitors of the PPP induce endodermal differentiation. (A) Double immunostaining Sox17/βIII-tubulin/DAPI of cells at 10 days of differentiation showed areas of immunoreactive cells for Sox17 in wt ES cells differentiated in presence of DHEA or 6AN. Scale bars, 50 µm. (B) qRT-PCR for Sox17 and GATA4 in wt ES cells at day 10 after treatment with DHEA or 6AN during neural differentiation. Values are means ± SD (n = 3). *P<0.05; **P<0.01; ***P<0.001.

Since both chemicals were able to inhibit the PPP in ES cells, we investigated their effect on wt ES cells differentiation. Immunofluorescence analysis revealed that both substances are able to induce differentiation of wt ES cells in Sox17+ cells (Figure 4A). Moreover, by qRT-PCR we observed an increase in the amount of GATA4 and Sox17 mRNA in DHEA and 6AN treated wt ES cells (Figure 4B).

## Discussion

Understanding how the endoderm forms from ES cells is the first step towards the ultimate goal, generating specific cell types for therapeutic purposes. Studies in *Xenopus laevis*, *zebrafish*, and mice collectively, suggest a conserved mechanism for mesoderm/endoderm lineage commitment involving the transforming growth factor-β (TGF β) family member Nodal, and a common set of downstream effector molecules [16], [17], [26].

One promising differentiation strategy is to recapitulate, *in vitro*, the developmental signals that guide cells towards specific lineages during development [19]. *In vitro* it has been shown that addition of Activin A or Nodal during ES cells differentiation leads to endodermal induction.

Recently, two groups [19], [27] illustrate high throughput screening to discover novel small molecules able to induce embryonic stem cell differentiation into definitive endoderm. However, the molecules reported have still necessity of serum presence in the differentiation protocols. This means that we are still not acquainted with all the pathways involved in endodermal differentiation and, moreover, we still don't know how to control them.

The PPP has been described to be essential in the cell during the defence against oxidative stress. Our results show, for the first time, that modulation of this metabolic pathway could influence stem cell differentiation. In fact, we observed that cells unable to produce pentose sugars through the PPP, under chemically defined conditions, spontaneously differentiate into endodermal precursor cells. In the same culture conditions, as we showed before [13], wt ES cells only differentiate into neuronal cells.

The specification of mesendodermal is postulated to be dependent on Tgf-β/Nodal pathway [16], [17]. Although Smad2 seems to be active also in wt ES cells, we observed an increased activation of this pathway in *G6pdΔ* ES cells; furthermore, expression of Cripto, the Nodal co-receptor, was persistent in *G6pdΔ* ES cells until day 6 of differentiation. These data suggest that mesendodermal differentiation could be dependent on Tgf-β/Nodal pathway in *G6pdΔ* ES cells. Moreover, modulation of the PPP seems to be required upstream Tgf-β/Nodal pathway activation during mesendodermal induction.

We showed that the mechanism implicated in this process involves the role of the PPP in the production of pentose sugars either than the previously described function in the oxidative stress defense. Indeed, we observed that reduction of oxidative stress, during the differentiation process in *G6pdΔ* ES cells, did not inhibit the Sox17 activation. Moreover, *Pgd*+/− ES cells, also having a deficit in the PPP, are able to generate endodermal precursor cells even if they have a normal resistance to oxidative stress due to the normal G6PD activity.

In contrast, addition of D-(-)-ribose, a pentose sugar produced by PPP, to the cell culture differentiation medium decreases the amount of Sox17 transcript, suggesting that the concentration of pentose sugars in the cells could be the signal that induces endodermal differentiation.

Furthermore, we identified two substances, DHEA and 6AN, known to inhibit the PPP, that act as endodermal inductors.

*G6pd* is an X-linked gene. In female heterozygous for G6PD mutation causing severe deficiency, once X inactivation has produced mosaicism for the G6PD cellular phenotype, there is a strong selection against G6PD(−) cells both in mouse and in human [12], [28]. Nevertheless, analysis of G6PD(+/−) heterozygous female showed that, differently from other tissues, intestinal crypts deriving each from an endodermal stem cell were severely G6PD deficient [12]. These data confirmed ours, in fact they suggested that also *in vivo* in absence of G6PD, cells show the intrinsic ability to colonize endodermal derived tissues and to differentiate into endodermal cells.

*Pgd* has been identified in ES cells as a direct target of Myc in two different ChIP-on-chip analysis [5], [29]. In a different experiment, cMyc has been described to induce the production of the pentose sugar [7]. Recent data has reported that genes of the PPP are among the most prominently induced by mTOR [6]. Inhibition of mTOR or simultaneous inactivation of c- and N-Myc induce endodermal differentiation [4], [5]. Our results raise the possibility that Myc and mTOR can repress endodermal differentiation activating the PPP.

The data described will help direct experiments aimed at ES cell differentiation into therapeutically relevant endodermal derivatives.

## Materials and Methods

### ES cell culture

AK7 (wt), E14 Tg2A (MMRRC; wt E14), *G6pdΔ*, *G6pdΔ* ^p*G6pd*^ and *Pgd*+/− (MMRRC Strain ID: 081091) ES cell lines were maintained in an undifferentiated state by culturing them on a mitomycin-C-inactivated fibroblast monolayer in presence of leukemia-inhibiting factor (LIF) [30]. Under these conditions the cell population remained undifferentiated, as determined by visual inspection under phase-contrast microscopy.

### In vitro differentiation

*In vitro* differentiation was performed according to Fico et al. (2008) [13]. Briefly, at 48h before inducing differentiation wt AK7, wt E14, *G6pdΔ*, *G6pdΔ* ^pG6pd^ and *Pgd*+/− ES cells were seeded on gelatin-coated plates. At day 0, ES cells were dissociated in a single-cell suspension and 1500 cells/cm^2^ were plated on gelatin-coated plates. The culture medium was replaced daily during differentiation process. Culture medium for neuronal differentiation (serum-free Knockout Serum Replacement (KSR)-supplemented medium) contained knockout Dulbecco minimal essential medium supplemented with 15% KSR (Invitrogen), 2 mM glutamine, 100 U/ml penicillin/streptomycin, and 0.1 mM β-mercaptoethanol.

Endoderm differentiation was performed adding 1.5 g/l of D-(-)-ribose in the differentiation medium. Addition of higher concentration of D-(-)-ribose during the differentiation induced cell death, lower concentration had no effect on endodermal differentiation.

To block the PPP we added DHEA and 6AN, at 100 µM and 10 µM final concentration respectively, in the differentiation medium starting from the plating and carrying on for the entire duration of the experiment.

### RNA isolation and RT-PCR

Total RNA was isolated through PerfectPure RNA Cultured Cell kit (5 PRIME). Reverse transcription-PCR (RT-PCR) was performed with the Perkin-Elmer RT-PCR kit, as recommended by the manufacturer. cDNA was amplified by PCR. The number of cycles was chosen to select PCR conditions on the linear portion of the reaction curve to avoid the saturation effects of PCR. Sequence of specific primers, number of cycles, annealing temperature, and the length of the amplified products have been reported in Table S1.

### Real-time RT-PCR

First-strand cDNA was synthesized from 500 ng of total RNA using oligo-dT primers, random hexamers and SuperScript II (Invitrogen). Real-time RT-PCR analysis was performed on Biorad CFX 96 Real time System using the SYBR Green PCR Master Mix (Biorad). The PCR reaction consists of 10 µl of SYBR Green PCR Master Mix, 120 ng of forward and reverse primers, and 4 µl of 1∶30 diluted template cDNA in a total volume of 25 µl and 40 cycles of amplification (95°C 10 s; 62°C 30 s; 72°C 10 s). Primer specificity was determined by melting curve analysis and standard curves were generated to check primer efficiency. The relative expression of each gene was normalized against GAPDH.

GATA4 forward 5′-CACTATGGGCACAGCAGCTCC-3′,

GATA4 reverse 5′-TTGGAGCTGGCCTGCGATGTC-3′;

Sox17 forward 5′-GGAGGGTCACCACTGCTTTA-3′,

Sox17 reverse 5′-AGATGTCTGGAGGTGCTGCT-3′;

Pdx1 forward 5′-TCACGCGTGGAAAGGCCAGT-3′,

Pdx1 reverse 5′-GTGTAGGCAGTACGGGTCCT-3′;

GAPDH forward 5′-TCTTCTGGGTGGCAGTGATG-3′,

GAPDH reverse 5′-TGCACCACCAACTGCTTAGC-3′;

Three independent PCR reactions were performed for any analyzed gene. Data were represented as mean ± SD of at least two independent experiments. Differences between control values and experimental values were compared by Student's *t* test.

### Immunocytochemistry

Cells were fixed in 4% paraformaldehyde and 1× phosphate-buffer saline (PBS) at room temperature for 30 min. Following fixation, samples were washed three times with 1× PBS for 5 min and then incubated with 10% normal goat serum (Dako Cytomation, Glostrup, Denmark, http://dakocytomation.com) and 0.1% triton X-100 in 1× PBS for 15 min at room temperature. The cells were then washed three times in 1× PBS for 5 min and incubated with primary antibodies (monoclonal anti βIII-tubulin, 1∶400, Sigma-Aldrich; polyclonal anti-GFAP, 1∶300, Dako Cytomation) in 10% normal goat serum and 1× PBS. For antibody anti-Sox17 and anti-GATA4 after fixation the cells were permeabilized with 0.5% triton X-100 in 1× PBS for 5 min, blocked with 0.1% Triton, 10% BSA and 1× PBS for 1 hr and incubated with primary antibody (goat polyclonal anti-Sox17, 1∶20, R&D; goat polyclonal anti-GATA4, 1∶100, Santa Cruz Biotecnology Inc.) in 0.1% triton, 10% BSA in 1× PBS at 4°C overnight. Following primary antibody incubation, cells were rinsed three times in 1× PBS and further incubated with secondary antibodies: either anti-mouse IgG FITC-conjugated (1∶400; Molecular Probe) or anti-rabbit IgG FITC-conjugated (1∶200; Santa Cruz Biotechnology) in 10% normal goat serum and 1× PBS in for 30 min at room temperature; anti-goat Alexa Fluor 594 (1∶400; Invitrogen) in 0.1% triton, 0,1% BSA for 30 min at room temperature. Finally, samples were washed three times in 1× PBS and counterstained with 4′, 6′-diamido-2-phenylindole (DAPI, 250 ng/ml; Sigma-Aldrich). Labelling was detected by fluorescent illumination using an inverted microscope (DMI 6000B, Leica Microsystems); images were acquired on a DCF 360 FX B/W camera (Leica).

### Western Blot Analysis

Cells were lysed in 1× RIPA lysis buffer in presence of protease inhibitor mixture (Roche)/1% phosphatase inhibitor mixture (Roche). Proteins were separated by 10% Tris-Glycine SDS/PAGE (Bio-rad) under denaturing conditions and transferred to a PVDF membrane. After blocking with 5% milk in 1× PBS/0.1% Triton X, the membrane was incubated with antibodies against phospho-Smad2 (1∶1000, Cell Signaling), Cripto (1∶1000), Olig2 (1∶1000, Dana Faber Cancer Institute), PARP (1∶1000, New England BioLabs) or β-actin (1∶1000 Cell Signaling) overnight at 4°C. The membrane was then washed, incubated with anti-mouse/rabbit peroxidase-conjugated secondary antibody (1∶1000, Cell Signaling) at room temperature for 1 hr, and developed by ECL plus (Amersham).

### Measurement of ^14^CO_2_ production

^14^CO_2_ produced by PPP or Glycolysis was determined as previously described [10]. Differences between control values and experimental values were compared by Student's *t* test.

### Measurement of ROS generation

ROS were detected using the fluorescent dye 2′,7′-dichlorofluorescein diacetate (DCFDA), (Molecular Probes, Eugene, OR) as previously described [31]. Differences between control values and experimental values were compared by Student's *t* test.

### Furosine Analysis

D-(-)-ribose treated and untreated *G6pdΔ* ES cells at day 13 of differentiation were lysed in water (32 µg/µl) and hydrolyzed in 8N hydrochloric acid (HCl) for 23 hr at 110°C. The hydrolysates were filtered through a 0.45 µm Whatman filter paper. A 0.5 mL aliquot of the filtered hydrolysate was purified by a C18 cartridge from which furosine was eluted by 3 mL of 3N HCl and 20 µL of the mixture was injected into the HPLC. Furosine was determined by ion-pair RP-HPLC as previously described [32]. The separation of furosine was performed in a C8 column (250×4.6 mm i.d.) (Alltech furosine- dedicated) (Alltech Associates, Laarne, Belgium).

## Supporting Information

Figure S1 **Evidence that GATA4+ and Sox17+ cells, formed during** ***G6pdΔ*** **ES cells differentiation, are endodermal precursors.** (A) Double immunostaining GFAP/GATA4 of cells at 13 days of differentiation show absence of co-localization between the two markers, indicating that GATA4 positive cells are not astrocytes. (B) Double immunostaining βIII-tubulin/GATA4 of cells at 13 days of differentiation show absence of co-localization between the two markers, indicating that GATA4 positive cells are not neurons. (C) Western blot analysis with anti-Olig2 and anti-Actin antibodies performed on protein extracts from wt and *G6pdΔ* undifferentiated ES cells (day 0) and at 10 days of neural differentiation. Actin was analyzed as loading control. (D–E) qRT-PCR for Nodal and Cripto in wt and *G6pdΔ* ES cells during differentiation. Values are means ± SD (n = 2). *P<0.05; **P<0.01; ***P<0.001.
(TIF)

Figure S2 **Differentiation in antioxidant conditions.** (A) Reduced amount of reactive oxygen species (ROS) is detected in *G6pdΔ* differentiated ES cells in presence of 5% oxygen compared with the ones cultured at 20% oxygen concentration. Values are means ± SD (n = 2). *P<0.05; **P<0.01; ***P<0.001. (B) RT-PCR of different lineage-specific markers in wt and *G6pdΔ* ES cells differentiated for 10 days in presence of NAC.
(TIF)

Figure S3 **Characteritazation of heterozygous knockout** ***Pgd*** **ES cells (** ***Pgd*** **+/−).** (A) RT-PCR analysis of *Pgd* mRNA level in undifferentiated *Pgd*+/− and wt E14 ES cells. Amplified HPRT is shown as a positive control. (B) Activity of the PPP determined by [1-^14^C] glucose and the cmp/mg of protein of ^14^CO_2_ released in wt and *Pgd+/−* ES cells. Values are means ± SD (n = 3). *P<0.05; **P<0.01; ***P<0.001. (C) wt, *G6pdΔ*, wt E14, and *Pgd+/−* undifferentiated ES cells were incubated with 0, 300 or 800 µM of Diamide, a thiol-oxidizing agent, for 30 min. After 8 hr, total proteins were extracted and separated on SDS-PAGE, and their respective content in cleaved PARP was analyzed by Western blotting. (D–E) Double immunostaining GFAP/GATA4 of wt E14 and *Pgd+/−* ES cells at 13 days of differentiation show absence of co-localization between the two markers, indicating that GATA4 positive cells are not astrocytes. (F) qRT-PCR for GATA4 in wt E14 and *Pgd+/−* ES cells during neural differentiation. Values are means ± SD (n = 3). *P<0.05; **P<0.01; ***P<0.001. (G) qRT-PCR for Sox17 in *G6pdΔ* ES cells at day 10 during neural differentiation in presence of different sugars: D-ribose (D-rib), L-ribose (L-rib), L-arabinose (L-arab) and sucrose (Sucr) at 10 mM final concentration. Values are means ± SD (n = 3). *P<0.05; **P<0.01; ***P<0.001.
(TIF)

Figure S4 **Characterization of ES cells treated with DHEA or 6AN.** (A) Activity of pentose phosphate pathway determined by 1-^14^C glucose and the cmp/mg of protein of ^14^CO_2_ released in wt ES cells treated with DHEA or 6AN. Values are means ± SD (n = 3). *P<0.05; **P<0.01; ***P<0.001. (B) ES cells treated with DHEA and 6AN were incubated with 300 µM of Diamide for 30 min. After 8 hr, total proteins were extracted and separated on SDS-PAGE, and their respective content in cleaved PARP was analyzed by Western blotting. Actin was analyzed as loading control.
(TIF)

Table S1 **Primers used and PCR conditions.**
(DOC)
